# Efficacy and safety of bortezomib maintenance in patients with newly diagnosed multiple myeloma: a meta-analysis

**DOI:** 10.1042/BSR20170304

**Published:** 2017-07-27

**Authors:** Chun-yan Sun, Jun-ying Li, Zhang-bo Chu, Lu Zhang, Lei Chen, Yu Hu

**Affiliations:** Institute of Hematology, Union Hospital, Tongji Medical College, Huazhong University of Science and Technology, Wuhan 430022, China

**Keywords:** bortezomib, maintenance therapy, meta-analysis, multiple myeloma

## Abstract

Multiple myeloma (MM) is a B-cell neoplasm with a high incidence of relapse. Bortezomib has been extensively studied for the maintenance treatment of MM. Here, we carried out a meta-analysis to determine the efficacy and safety of maintenance therapy with bortezomib. We searched for clinical trials in PubMed (Medline), Embase (OVID), and the Cochrane Library. Two randomized controlled trials (RCTs) enrolling a total of 1338 patients were included. Bortezomib maintenance statistically significantly improved both progression-free survival (PFS) (hazard ratio (HR) 0.67, 95% confidence interval (CI) = 0.51 to 0.87, *P*=0.003) and overall survival (OS) (HR = 0.75 therapy, 95% CI = 0.63 to 0.89, *P*=0.001) more than did non-bortezomib maintenance therapy. Our analysis revealed higher incidence of neutropenia (risks ratios (RR) = 1.39; 95% CI = 1.08 to 1.79), peripheral neuropathy (PN) (RR = 2.23; 95% CI = 1.38 to 3.61, *P*=0.001), and cardiologic events (RR = 1.91; 95% CI = 1.12 to 3.28, *P*=0.02) in patients with bortezomib maintenance therapy. Our meta-analysis demonstrates OS and PFS benefits of bortezomib maintenance therapy in patients with newly diagnosed MM. However, the therapy is associated with increased risk of adverse events. Additionally, more RCTs are needed for better understanding and determination of optimal bortezomib maintenance therapy in MM.

## Introduction

Multiple myeloma (MM), a disease results from a proliferation of plasma cells and thus characterized by an elevation in immunoglobulin, is the second most frequent hematologic malignancy around the world. The median age at diagnosis is 70 years, with 37% of them younger than 65 years old, 26% aged from 65 to 74 years, and 37% beyond 75 years. The incidence rates in men are higher than in women [1,2]. The application of high dose therapy (HDT) and autologous stem cell transplantation (ASCT) as well as the advent of novel agents (e.g. immunomodulatory drugs including thalidomide and lenalidomide, and the proteasome inhibitor bortezomib) improve survival in MM but the disease still remains incurable due to high incidence of relapse. Therefore, MM maintenance therapy, a treatment given for a specified duration to maintain the response of first-line therapy and prolong survival [3], is of great interest to clinical and translational researchers.

Early trials incorporating conventional chemotherapy, interferon, or glucocorticosteroids into maintenance therapy failed to show satisfactory results due to limited survival benefit or toxicity [4]. Three meta-analyses evaluating thalidomide maintenance therapy showed progression-free survival (PFS) and overall survival (OS) benefits in transplantation-eligible patients [5,6]. However, thalidomide maintenance has several limitations, including the toxic risk of peripheral neuropathy (PN), shorter OS in patients with high-risk cytogenetics [7], and less obvious improvement in OS for elderly patients [8–11]. Clinical trials using another immunomodulatory drug lenalidomide for maintenance therapy showed effectiveness in response rates and PFS, but also treatment-related adverse events and potential risk of second primary malignancies (SPMs) [12,13].

Bortezomib is a boronic acid-based reversible proteasome inhibitor involving in the ubiquitin–proteasome pathway of cellular protein homeostasis. Disruption of proteasome activity results in cell growth arrest and apoptosis. Malignant plasma cells in MM produce large amount of immunoglobulins and have higher levels of proteasome activity compared with normal cells. Therefore, MM cells are more sensitive to the pro-apoptotic effects of proteasome inhibition than normal cells [14,15]. Bortezomib-based induction therapy has already shown improved PFS and OS, even for those patients with *t* (4; 14) or renal failure [16,17], and therefore is recommended for both transplantation-eligible and transplantation-ineligible newly diagnosed MM patients [18]. This leads to further investigation for incorporating bortezomib into maintenance phase. To obtain a better understanding of the efficacy and safety of bortezomib-based maintenance therapy in newly diagnosed MM patients, we carried out this meta-analysis.

## Methods

### Article inclusion/exclusion criteria and quality

We searched for clinical trials in PubMed (Medline), Embase (OVID), and the Cochrane Library using key words ‘myeloma’, ‘bortezomib OR Velcade’ and ‘maintenance OR consolidation OR continuous therapy OR continuous treatment’. To identify eligible studies that may have been missed during the initial online search, we further examined the reference lists of relevant reviews and trials identified. The last search dated back to November, 2015.

Two investigators independently reviewed all the titles and abstracts obtained from the above search strategy. Potentially related articles were then checked in full text to identify phase III randomized controlled trials (RCTs) that compared the outcomes of bortezomib-based and non-bortezomib-based maintenance therapies in newly diagnosed MM patients. Included studies were required to report PFS and OS. Duplicated studies were regarded as one.

Two investigators independently evaluated the methodological quality (i.e. the randomization, blinding method, and completeness of follow-up) of the included studies using the Jadad scale, which could show us intuitive results by giving each study a score. Scores 3–5 and 0–2 were associated with high and low quality respectively [19]. Additionally, we checked if these studies had adopted intention to treat (ITT) analysis and reported allocation concealment, considering the neglect in Jadad scale [20].

### Statistical analysis

Revman software (5.3) was used to perform all calculations related to meta-analysis. PFS was measured from the date of randomization to the time of disease progression, relapse, or death. OS was calculated as the time from randomization until death from any cause. We used hazard ratio (HR) with 95% confidence interval (95% CI) of OS and PFS outcomes for the bortezomib maintenance treatment arm over the non-bortezomib treatment arm to evaluate the efficacy. Dichotomous outcomes about adverse effects were evaluated using risks ratios (RR) with 95% CIs. Pooled results of HR and RR were calculated based on the inverse variance (IV) method and the Mantel–Haenszel (M–H) method respectively. Statistical heterogeneity was assessed using the *I*^2^ test, and the DerSimonian and Laird random effects model was applied when heterogeneity was significant (*I*^2^>50%) [21,22]. The publication bias assessment was not formally carried out due to limited number of included trials.

## Results

### Selection of studies

We identified 498 publications through initial search and kept 22 of them for further full-text review after title and abstract screening. Nineteen publications were excluded after full-text review and only three articles [23–25] were remained to our final analysis. It is noted that two articles [24,25] providing important data from one trial were considered as one in our analysis. A phase III PETHEMA/GEM randomized trial comparing patients who received maintenance therapy after induction and ASCT with either interferon-α or thalidomide or thalidomide plus bortezomib was included at the beginning but excluded at last due to lack of sufficient data for analysis [26]. Therefore, finally two RCTs were included in the present meta-analysis (Figure 1).

**Figure 1:** Flow diagram of study selection.

The characteristics of the two trials are summarized in Table 1. One study published in 2014 was conducted at 61 centers in Italy from May, 2006 to January, 2009 [23]. A total of 511 newly diagnosed myeloma patients who were not candidates for high-dose therapy plus stem-cell transplantation (age >65 years or with coexisting comorbidities) were randomly assigned to receive VMPT (melphalan, prednisone, bortezomib, thalidomide) induction plus VT (bortezomib, thalidomide) maintenance (254 patients) or VMP (melphalan, prednisone, bortezomib) induction without maintenance (257 patients) for 2 years. The median age is 71 years and median follow-up time is 54 months. The other study, conducted by the Dutch-Belgian Hemato-Oncology Cooperative Group (HOVON) and the German Multicenter Myeloma Group (GMMG), was published in 2012 as full text, and its extended follow-up was reported as abstract in 2013 [24,25]. A total of 827 eligible, newly diagnosed, symptomatic MM patients were randomly assigned to VAD (vincristine, doxorubicin, dexamethasone) induction intensification with high-dose melphalan (HDM) and ASCT-thalidomide maintenance (arm A, 414 patients) or PAD (bortezomib, doxorubicin, and dexamethasone) induction intensification with HDM and ASCT-bortezomib maintenance for 2 years (arm B, 413 patients). The median age is 57 years and median follow-up time is 67 months.

**Table 1:** Characteristics of studies included in the meta-analysis

Study	People	*N*	Maintenance therapy regimen	Planned maintenance duration	Median follow-up	Median PFS
Sonneveld, P. (2013) (HOVON-65/GMMG-HD4)	Eligible, newly diagnosed, symptomatic MM	827	Arm A (*n*=414): daily thalidomide 50 mg	2 years	67 months	N/A
	Median age: 57		Arm B (*n*=413): 2-weekly bortezomib 1.3 mg/m^2^ i.v.			
Palumbo, A. (2014) (Italy)	Newly diagnosed, not candidates for HDM + ASCT	511	VT (*n*=254); No maintenance (*n*=257)	2 years	54 months	VMPT-VT: 35.3 months
	Median age: 71					VMP : 24.8 months

Abbreviations: ASCT, autologous stem cell transplantation; N/A, not available; VMP, bortezomib–melphalan–prednisone; VMPT-VT, bortezomib–melphalan–prednisone–thalidomide followed by maintenance with bortezomib–thalidomide; VT, bortezomib at a dose of 1.3 mg/m^2^ every 15 days and thalidomide at a dose of 50 mg per day.

The methodological quality of the included studies is shown in Table 2 with Jadad scale. Additionally, both studies applied ITT analysis (ITT) and neither of them offered any information about allocation concealment.

**Table 2:** Quality score of included studies applying Jadad scale

Study	Randomization	Blinding	Lost/Withdrawal to follow-up	Total
Sonneveld, P. (2013) (HOVON-65/GMMG-HD4)	2	0	1	3
Palumbo, A. (2014) (Italy)	1	0	1	2

### Efficacy

The pooled HR of PFS was 0.67 (95% CI = 0.51 to 0.87, *P*=0.003), indicating a trend of PFS improvement with bortezomib maintenance. However, there was a significant heterogeneity between the two trials (*P*=0.05, *I*^2^ = 74%, Figure 2). The pooled HR of OS shows the bortezomib maintenance therapy arm is superior (HR = 0.75, 95% CI = 0.63 to 0.89, *P*=0.001). No significant heterogeneity was revealed between the two trials (*P*=0.56, *I*^2^ = 0%, Figure 3).

**Figure 2:** Pooled HRs of PFS comparing bortezomib maintenance therapy arm with non-borzomib maintenance therapy arm.

**Figure 3:** Pooled HRs of OS comparing bortezomib maintenance therapy arm with non-borzomib maintenance therapy arm.

### Safety

Both trials have reported the incidence of adverse events. So, we carried out a meta-analysis measuring pooled RR to compare grade 3–4 adverse events in bortezomib maintenance therapy arm and non-bortezomib maintenance therapy arm. The analysis revealed significant differences between the two arms, and the bortezomib maintenance therapy statistically showed significantly increased risk for developing neutropenia (RR = 1.39; 95% CI = 1.08 to 1.79), PN (RR = 2.23; 95% CI = 1.38 to 3.61, *P*=0.001), and cardiologic events (RR = 1.91; 95% CI = 1.12 to 3.28, *P*=0.02) (Figure 4). We did not observe a significant difference in the risk of developing anemia, thrombocytopenia, infection, deep vein thrombosis and gastrointestinal (GI) symptoms between the two arms. No evidence of significant heterogeneity was revealed between the two trials.

**Figure 4:** Pooled RR of grade 3–4 adverse events comparing bortezomib maintenance therapy arm with non-bortezomib maintenance therapy arm: Different events are separately shown from subparts (a) to (h) (**a**) Neutropenia, (**b**) thrombocytopenia, (**c**) anemia, (**d**) infection, (**e**) deep vein thrombosis, (**f**) PN, (**g**) cardiologic events, and (**h**) GI symptoms.

## Discussion

During the past decade, bortezomib has been shown to have great benefit in induction therapy of MM patients, thus leading to further clinical trials incorporating bortezomib into maintenance therapy. The objective of an ideal maintenance therapy is to improve PFS and OS with minimal toxicity and without interfering patients’ quality of life [3]. Therefore, we carried out this meta-analysis to evaluate the efficacy and safety of bortezomib maintenance in MM.

Two RCTs with a total of 1338 patients were included in our analysis. Both significant PFS and OS improvement were seen in our pooled results with bortezomib maintenance over non-bortezomib maintenance therapy. This result indicates the benefit of bortezomib during maintenance in MM patients. Notably, according to an analysis of PFS calculated from the time of last HDM in HOVON-65/GMMG-HD4 trial, a significant difference in favor of the PAD arm was observed, indicating that although post-transplantation bortezomib and thalidomide both achieved response upgrades, bortezomib contributed more to improvement of PFS [24]. It is noted that a significant heterogeneity exists when calculating the pooled HR results of PFS. We considered that the heterogeneity comes from several sources. First, the different characteristics of individual patients in two studies could affect the evaluated results, including age, coexisting comorbidities, or MM severity. Second, both the induction and maintenance regimes differed between the two studies. Furthermore, we should take measurement bias into consideration.

Regarding the safety of applying bortezomib during maintenance, our analysis revealed significant differences between the two arms. Higher incidence of neutropenia, cardiologic events, and PN were observed in patients of the bortezomib maintenance group. Consistent with previous reports, PN is the most frequent adverse effect, which could be managed by dose adjustment, subcutaneous administration, and decreasing the frequency of administration of bortezomib (Millennium Pharmaceuticals, Inc. VELCADE^®^ (bortezomib) official website http://www.velcade.com/Treatment-with-velcade/Possible-side-effects (2016)) [27]. As for supplementary specification, newly developed grade 3–4 PN occurred in 8% of patients during thalidomide maintenance and 5% of patients during bortezomib in HOVON-65/GMMG-HD4 trial, and for VMPT-VT arm in the study of Palumbo et al. [23] containing both bortezomib and thalidomide during maintenance the incidence of PN was 11% [24].

However, conflicting results have also been reported in other studies. A phase III PETHEMA/GEM randomized trial compared bortezomib/thalidomide, thalidomide, and Alfa2b-interferon as maintenance therapy after stem-cell transplantation for MM patients for a median follow-up of 34.9 months. The results showed that the PFS was significantly longer with TV compared with the other two arms (*P*=0.0009), but there was no significant difference in OS among the three arms [26]. In the UPFRONT study with patients’ median age higher than 70 years comparing VD, VTD, and VMP induction followed by bortezomib maintenance, only 5% of patients experienced grade ≥3 PN during maintenance, without adverse influence on patients’ quality of life [28,29].

In addition, the GEM2005MAS65 randomized trial investigated by the Spanish myeloma group compared maintenance therapy with bortezomib plus thalidomide (VT) or prednisone (VP) in elderly untreated myeloma patients, who had previously received induction with bortezomib, melphalan, and prednisone or bortezomib, thalidomide, and prednisone. The results showed an increase in complete response (CR) rate, remarkably long PFS, and acceptable toxicity, suggesting clinical benefit of bortezomib-based maintenance therapy [30]. Another analysis of the phase III HOVON-65/GMMG-HD4 trial showed that the known adverse impact of deletion 17p (del17p13) can be markedly reduced by incorporating bortezomib into the treatment and may be important for the long-term management of patients with this high-risk feature [31].

In view of the facts mentioned above, we suggest that more RCTs are needed to help us further understand the efficacy and safety of bortezomib maintenance in MM with different characteristics of patients and diverse drug combination regimes.

Our analysis was carried out through a standardized process, but it also has some limitations. First, only two studies were included in our analysis after comprehensive search and careful selection. One study without sufficient data was excluded [26]. Second, possible publication bias can affect our interpretation. Third, the Italian study didn’t report proper techniques for randomized allocation. And in both studies, randomized allocation were applied only before induction but not maintenance therapy, which led to difficulty in making a clear dissection of the role of bortezomib maintenance therapy. Fourth, due to the paucity of studies, we couldn’t perform a sensitivity analysis. In addition, variant characteristics of patients enrolled in the two RCTs, different study designs and varied length of follow-up time may also influence the statistical power of pooled outcomes.

In conclusion, our meta-analysis showed significant OS and PFS benefits of bortezomib maintenance therapy in patients with newly diagnosed MM. However, the increased risk of adverse events warrants serious consideration and adequate measures. Future RCTs are needed for better understanding and optimizing bortezomib maintenance therapy in MM.

## Abbreviations

ASCT: autologous stem cell transplantation
CI: confidence interval
HDM: high-dose melphalan
HDT: high dose therapy
HR: hazard ratio
IV: inverse variance
MM: multiple myeloma
OS: overall survival
PFS: progression-free survival
PN: peripheral neuropathy
RR: risks ratios
SPM: second primary malignancy
